RETRACTED

# The Survival Benefit of Liver Transplantation for Hepatocellular Carcinoma Patients with Hepatitis B Virus Infection and Cirrhosis

**DOI:** 10.1371/journal.pone.0050919

**Published:** 2012-12-07

**Authors:** Qing Zhang, Xinguo Chen, Yunjin Zang, Li Zhang, Hong Chen, Letian Wang, Yujian Niu, Xiuyun Ren, Zhongyang Shen, Lei Shang

**Affiliations:** 1 Institute of Liver Transplantation, General Hospital of Chinese People's Armed Police Force, Beijing, China; 2 Department of Health Statistics, Faculty of Preventive Medicine, Fourth Military Medical University, Xi'an, China; 3 First Department of Surgery, Shaanxi Provincial Corps Hospital of Chinese People's Armed Police Force, Xi'an, China; Drexel University College of Medicine, United States of America

## Abstract

**Background:**

A precise predictive survival model of liver transplantation (LT) with antiviral prophylaxis for hepatitis B virus (HBV)-associated hepatocellular carcinoma (HCC) and cirrhosis has not been established. The aim of our study was to identify predictors of outcome after LT in these patients based on tumor staging systems, antitumor therapy pre-LT, and antiviral prophylaxis in patients considered to be unfit by Milan or UCSF criteria.

**Methods:**

From 2002 to 2008, 917 LTs with antiviral prophylaxis were performed on patients with HBV-cirrhosis, and 313 had concurrent HCC.

**Results:**

Stratified univariate and multivariate analyses demonstrated that independent predictors for poor survival were tumor size >7.5 cm (P = 0.001), tumor number >1 (P = 0.005), vascular invasion (P = 0.001), pre-LT serum alpha-fetoprotein (AFP) level ≥1000 ng/ml (P = 0.009), and pre-LT aspartate aminotransferase (AST) level ≥120 IU/L (P = 0.044). Pre-LT therapy for HCC was an independent predictor of better survival (P = 0.028). Based on CLIP and TNM tumor staging systems, HCC patients with HBV-cirrhosis who met the following criteria: solitary tumor ≤7.5 cm, or ≤4 multifocal nodules, the largest lesion ≤5 cm and total tumor diameter ≤10 cm, or more nodules with the largest lesion ≤3 cm, and pre-LT serum AFP level <1000 µg/L and AST level <120 IU/L without vascular invasion and lymph node metastasis who were unfit for UCSF, had survival rates of 89% at 5 years. There was a 47% 5-year survival rate for patients with HCC exceeding the revised criteria.

**Conclusions:**

The current criteria for LT based on tumor size, number and levels of AFP and AST may be modestly expanded while still preserving excellent survival after LT. The expanded criteria combined with antiviral prophylaxis and pre-LT adjuvant therapy for HCC may be a rational strategy to prolong survival after LT for HCC patients with HBV-associated cirrhosis.

RETRACTED

## Introduction

Hepatitis B is endemic to China [1]. Of the 350 million individuals worldwide infected with the hepatitis B virus (HBV), one-third resides in China, with 130 million carriers and 30 million chronically infected people [2], [3]. The chronically infected individuals may be either asymptomatic or have chronic inflammation of the liver that leads to cirrhosis over a period of several years. HBV infection dramatically increases the incidence of hepatocellular carcinoma (HCC), the most common primary malignant cancer of the liver [4]. Furthermore, HBV-induced cirrhosis (HBV-cirrhosis) is the most common cause of HCC. In China, most HCC patients also have HBV-related cirrhosis [5].

The relationship between HCC with HBV-associated cirrhosis has long been recognized, and the primary therapeutic modality for HCC is surgical extirpation. Unfortunately, only a small number of patients are suitable for liver resection because of the advanced stage of tumors at the time of diagnosis, as well as the frequent development of tumors in a background of HBV-associated cirrhosis with poor liver function.

It has been established that liver transplantation (LT) with antiviral prophylaxis is the only therapeutic option for simultaneously treating HCC and HBV-associated cirrhosis [6]–[9], and it is accepted that LT is superior to hepatic resection in early HCC with cirrhosis [10]–[13].

Mazzaferro et al. reported good LT outcomes for small HCC ([Milan] criteria: (solitary tumor ≤5 cm, or three or fewer lesions none >3 cm) with cirrhosis, with 4-year overall and recurrence-free survival rates of 85% and 92%, respectively [8]. Recently, a set of expanded criteria for tumor staging was proposed that was associated with excellent survival after OLT. HCC patients who met UCSF criteria (solitary tumor ≤6.5 cm or 3 nodules with the largest lesion ≤4.5 cm, and a total tumor diameter ≤8 cm) after LT had 1- and 5-year survival rates of 90% and 75.2%, respectively [14], which were similar to the survival rates in patients without HCC. Nevertheless, for patients with HBV-associated HCC, there are usually more aggressive tumors and elevated hepatitis activity that could lead to hepatocyte necrosis, as well as HBV-associated cirrhosis with poor liver function. Despite several criteria showing excellent outcomes for LT for HCC [6], [8], [15]–[17], those criteria only focused on the size and number of tumors or pathologic tumor staging. They did not consider HCC induced by various other etiologies, other tumor factors, or liver markers, such as pre-LT serum alpha-fetoprotein (AFP) levels, Child-Pugh scores or liver function indicators, as determinants of HCC patient outcome. Nevertheless, there is no clear consensus for HBV-associated HCC, especially for advanced HCC patients with HBV- cirrhosis who may still have a favorable outcome after LT.

RETRACTED

Factors affecting outcome in patients with aggressive HCC have been extensively studied [14], [18], [19]. It has been shown that tumor size, tumor number, pathologic tumor differentiation, the presence or absence of vascular invasion, lymph node metastases, pre-LT serum alpha-fetoprotein (AFP), liver function lever, and preoperative tumor treatment are prognostic variables that have a clear impact on outcome [7], [8], [14], [20]–[22]. Tumor TNM staging for predicting survival of HCC patients has also been considered in the past. Recently, some studies [23], [24] have claimed that the Cancer of the Liver Italian Program (CLIP) staging system is one of the best staging systems in predicting survival in patients with advanced HCC compared to the Japanese, and AJCC TNM, and TNM sixth edition. The others lacked any prognostic parameters of liver dysfunction or AFP. A staging system that combines tumor factors, tumor marker(s) and hepatic function is the best predictor of prognosis of HCC patients, especially for HCC with HBV-associated cirrhosis. Some studies have reported that tumor diameter, poor tumor differentiation, vascular invasion, AFP level, HBV reinfection and prophylaxis were independent predictors of outcome [18], [25], [26].

Although most studies have shown that HBV infections carry a high risk of recurrence after resection or LT [27], prophylactic use of hepatitis B immunoglobulin (HBIG) combined with the nucleoside analogue lamivudine can markedly decrease the reinfection rate of HBV by suppressing HBV replication [28], [29]. Some reports have demonstrated that dual prophylaxis for HBV after LT reduces the risk of HBV reinfection and improves patient survival [30]. Therefore, it is possible that a subset of HBV-associated HCC patients who exceed Milan or UCSF criteria may still have a favorable outcome after LT.

In patients with HBV-related HCC, the tumors are usually large and aggressive and accompanied by elevated inflammatory activity that can lead to aggressive hepatocyte necrosis. In spite of the proposed expanded criteria such as UCSF [31], Pittsburgh [31] or UNOS to select HCC patients for LT [32], no universally accepted criteria have been established to select suitable HCC patients with HBV-cirrhosis for LT. The aim of this study was to establish criteria to select suitable HCC patients with HBV-cirrhosis for LT with antiviral prophylaxis and anti-HBV treatment.

## Materials and Methods

### Patient population

Between July 2002 and December 2008, 917 LTs with antiviral prophylaxis were performed for HBV cirrhosis at the Institute of Liver Transplantation, General Hospital of Chinese People's Armed Police Force, China (according to the China Liver Transplant Registry: https://www.cltr.org/). Of these 917 patients, 313 patients who were diagnosed with HCC and HBV-induced cirrhosis, underwent LT and had complete follow up information were enrolled in this study. HCC patients with extra-hepatic tumor metastasis, including lymph node metastasis or inferior vena cava tumor thrombus by imaging diagnosis before LT, were excluded from this study. Because the majority of cases who exceeded the Milan or UCSF criteria without tumor downgrading therapy pre-LT had been transplanted before 2004, the cases with a total tumor diameter of tumor nodules >12 cm were excluded from this study. In addition, patients with HBV co-infection with hepatitis C were also excluded from this study. The baseline characteristics of the 313 patients are summarized in Table 1.

RETRACTED

**Table 1:** The main clinical and pathological characteristics of the study patients.

Variables	N (%)
Gender	
Male	288 (92.0)
Female	25(8.0)
Age (year)	
≤50	151(48.2)
>50	162(51.8)
HBeAg	
Negative	204(65.2)
Positive	109(34.8)
HBV-DNA (×10^3^ IU/ml)	
<1	118(37.7)
<2500	145(46.3)
≥2500	39 (96.5)
Child-Pugh score	
A	118(37.7)
B	131(41.9)
C	64(20.4)
ALT (IU/L)	
1N,	134(42.8)
≥1N, <2N	104(33.2)
≥2N, <3N	37(11.8)
≥3N	38(12.1)
AST(IU/L)	
1N,	104(33.2)
≥1N, <2N	116(37.1)
≥2N, <3N	47(15.0)
≥3N	46(14.7)
ALP(IU/L)	
1N,	204(65.2)
≥1N, <2N	85(27.2)
≥2N	24(7.7)
Tumor size (cm)	
≤3	115(36.7)
>3, ≤5	121(38.7)
>5, ≤7.5	40(12.8)
>7.5	37(11.8)
Number of tumor nodules	
Single	214(68.4)
2	56(17.9)
3	15(4.8)
4,	5(1.6)
>4	23(7.3)
Tumor differentiation	
I (well)	13(4.2)
II (moderate)	278(88.8)
III (poor)	22(7.0)
Serum AFP level (ng/ml)	
≤500	247(84.0)
500–1000	16(5.1)
1000–2000	23(7.3)
2000–5000	15(4.8)
≥5000	12(3.8)
Venous invasion	
Absent	272(86.9)
Present	41(13.1)
Lymph node invasion	
Absent	295(94.2)
Present	18(5.8)
Pre-LT antitumor therapy	
Absent	48(15.3)
Present	96(30.7)
Fit Milan criteria?	
Yes	179(57.2)
No	134(42.8)
Fit UCSF criteria, but unfit Milan?	
Yes	42(13.4)
No	271(86.6)
Post-LT HBsAg reinfection	
Negative	293(93.6)
Positive	20(6.4)
Rejection	
Absent	285(91.1)
Present	28(8.9)
Post-LT treatment for recurrence	
Absent	259(82.7)
Present	54(17.3)

In the current study, there were 288 men and 25 women, aged 25 to 70 years, with a median age of 49.65 years. The mean tumor size was 4.37 cm (±2.7, range 0.3–12.0). AFP levels and liver function indicators were obtained within 1 month before LT. The median AFP level was 1,016 µg/L (range 1.62 to 60,500 µg/L). The median ALT, AST and ALP level were 93.8 IU/L (range 8 to 3196 IU/L), 109.7 IU/L (range 17 to 4409 IU/L) and 114.8 IU/L (range 23 to 643 IU/L), respectively. Of the 313 patients, 122 (38.9%) had normal AFP levels (<20 IU/L). HBV DNA levels obtained within 3 months before OLT were available in 302 of 313 patients. The median HBV DNA level was 2,500 IU/ml (range, 11.4–91200). All patients were tested positive for HBsAg.

RETRACTED

In addition, 96 of 313 patients were given pre-LT treatments: 82 cases of transarterial chemoembolization, of which 4 were combined with percutaneous ablations and 7 were followed with hepatic resection, 8 cases of percutaneous ablations with radio frequency, 2 percutaneous ablation cases with ethanol injection, and 10 resection only cases before LT (when there was intrahepatic recurrence of hepatocellular carcinoma). No tumor adjuvant treatment was given after LT unless tumor recurrence was detected.

In an additional analysis, the entire cohort of 313 patients with HCC were divided into 3 groups: 197 (57.2%) fit the Milan criteria group, 42 (13.4%) did not fit the Milan, but did fit the UCSF criteria (Milan-UCSF) group, and 92 (29.4%) in the group with patients who exceeded UCSF criteria(>UCSF), of which 38 (41.3%) were given pre-LT treatments for downgrading therapy or decreasing the risk of tumor dissemination during the long waiting period for LT.

This retrospective study was performed incompliance with principles of the Helsinki Declaration, and institutional guidelines.

### Diagnosis and evaluation

As a part of the pre-transplant workup for HBV in recipients, infection with HBV pre-LT was routinely checked by the following viral markers: hepatitis B surface antigen (HBsAg), antibody to HBsAg (anti-HBs), hepatitis B core antibody, hepatitis Be antigen (HBeAg), and hepatitis B virus deoxyribonucleic acid (HBV DNA) levels. Pre-transplant HBV infection was defined as serum HBsAg and/or HBV DNA positivity. HBV status was assessed before and after transplantation with HBV markers detection and HBV DNA PCR assay. Tests to determine viral mutation were also conducted to identify resistance to lamivudine or adefovir. In order to differentiate HBV recurrence from graft rejection, a percutaneous or transjugular liver biopsy was performed.

HCC was diagnosed pre-LT by measuring serum AFP levels, and by a combination of 2 abdominal imaging techniques (ultrasound, computed tomography [CT], positron emission tomography [PET], or magnetic resonance imaging [MRI]). Final diagnosis of HCC and cirrhosis in the explanted livers was determined by pathological examination. Routine post-LT examinations included abdominal ultrasonography, X-ray imaging, serial serum AFP levels, and whole-body CT scans, as deemed necessary. During LT follow-up, early tumor recurrence or metastasis was assessed by AFP level and abdominal ultrasonography once a month by whole-body CT or MRI examinations, and by bone scintigraphy every 3–6 months. To histologically confirm recurrence, a biopsy was conducted if necessary. Liver function was routinely checked pre-LT and post-LT.

RETRACTED

The explanted livers were fixed in formalin and examined by two experienced pathologists. The number of tumors, tumor size (maximum diameter of tumor nodules), the presence of vascular invasion, perihepatic lymph node invasion, and the degree of differentiation (well, moderately, and poorly differentiated) were recorded.

The total tumor diameter for patients with multiple tumor nodules was calculated as the sum of the maximal diameter of each lesion. The total tumor diameter could not be calculated in patients with numerous tumor nodules too small to measure. Three hundred and thirteen patients were identified and were staged using tumor staging systems: the Cancer of the Liver Italian Program (CLIP) and TNM classification (UICC/AJCC,2010) [23]. The pathologic tumor stage (T) was determined according to the TNM staging system. For patients with known solitary or multicentric tumors detected by two imaging methods, tumor size was calculated using tumor nodules identified in the liver explants.

### Antiviral protocols

All patients were routinely given hepatitis B immunoglobulins and nucleoside analogues (lamivudine, adefovir, or entecavir) based on the antiviral protocol shown in Table 2.

**Table 2:** Antiviral prophylaxis for HBV reinfection after LT.

Patients with high risk of HBV reinfection	Patients with low risk of HBV reinfection
(HBV-DNA ≥105 copies/ml, or HBeAg [+])	(HBV-DNA <105copies/ml, or HBeAg[−])
**Pre-LT:** nucleoside analogues, qd 2–4w	**Pre-LT:** nucleoside analogues, qd 0–2 w
**Intraoperative:** HBIG 4000 IU, iv	**Intraoperative:** HBIG 2000 IU, iv
**Post-LT:** HBIG 1000 IU, iv, qd, 1–7d	**Post-LT:** HBIG 1000 IU, iv, qd, 1–7d
After 7 days, HBIG 1000 IU, iv, once a week; or HBIG 400 IU, im, qd or qod or twice a week	After 7 days, HBIG 1000 IU, iv, once a week; or HBIG 400IU, im, qd or qod or twice a week
Adjust frequency of HBIG administration to reach target therapeutic concentration	Adjust frequency of HBIG administration to reach target therapeutic concentration.
**Target therapeutic concentration Post-LT**	**Target therapeutic concentration Post-LT**
≤6 months post-LT: anti-HBs titre ≥500 IU/L	≤6 months post-LT: anti-HBs titre ≥300 IU/L
6–12 months post-LT: anti-HBs titre ≥200 IU/L/	6–12 months post-LT: anti-HBs titre ≥200 IU/L
≥12 months post-LT: anti-HBs titre ≥100 IU/L	≥12 months post-LT: anti-HBs titre ≥100 IU/L

RETRACTED

### Immunosuppressive therapy

During LT, all patients were administered a drug regimen based on the calcineurin-inhibitor combined with mycophenolate mofetil (MMT) and prednisone. Prednisone was gradually withdrawn within 3 months after LT, and sirolimus was initiated 3 months after LT. During follow-up, patients were given long-term treatments with tacrolimus or cyclosporin A alone or combined with either MMT or sirolimus.

### Statistical analysis

Overall and disease/recurrence-free survival analyses were performed with the Kaplan-Meier method, and the survival time was calculated from the day of operation to either the day of death or the most recent follow-up visit. Group survival curves were compared using the log-rank test (Mantel-Cox). Clinical variables and univariate correlations between overall survival and recurrence-free survival were determined using the Chi-square test and the Spearman rank test, respectively. In addition, all variables were analyzed for independent significance using multivariate step-wise Cox regression analysis. Statistical calculations were performed by SPSS 11.0 statistical software. The significance level was defined as two-sided (P<0.05).

## Results

In the study, 313 adult LT patients with HBV-associated HCC and cirrhosis had complete follow-up. The median follow-up period was 65.0 months (61.9±28.3; range 2–120). The main clinical and tumor pathology characteristics of the 313 patients are shown in Table 1.

After LT, 20 of the 313 patients (6.40%) were found to have been re-infected with HBV hepatitis (20 cases were serum HBsAg positive, 6 were HBeAg positive, and 14 were HBV DNA probe positive). Thirteen of 20 patients had HBV reinfection, of which 4 were withdrawn from antiviral prophylaxis due to HCC occurrence, 2 were withdrawn by themselves without doctor's orders, and 7 patients were withdrawn from hepatitis B immune globulin treatment (HBIG) 2 years after LT.

### Histologic Data and Tumor Staging Systems

The pathologic tumor characteristics of 313 HCC patients based on the TNM classification (sixth edition; T1-4 stage) and CLIP tumor staging systems are summarized in Table 3. One-hundred and forty of the 313 (44.8%) patients had CLIP 0 or 1, of which 125 had solitary lesions ranging from 1 to 7 cm in diameter, and 15 were multifocal tumor lesion (no more than 3 lesions). In 178/313 (56.9%) patients at stage T1 had solitary lesions of 4.16 cm (±2.329) in diameter. In 82/313 (26.2%) patients with CLIP 2, 43 tumors were solitary, 36 were multifocal tumor lesions (≤4 tumor lesions), and 3 had >4 tumor nodules, while in 85/313 (27.2%) patients at stage T2 with tumor sizes ≤5 cm, 6 tumors were solitary, 61 were multifocal tumor lesions (≤4 tumor lesions), and 18 had >4 tumor nodules. In 51/313 (16.3%) patients with CLIP3, 23 were solitary, 20 were multifocal lesions (≤4 tumor lesions), and 8 had >4 tumor nodules. In 32/313 patients (10.2%) at stage T3 with a median tumor size of 7.58 cm (±3.234) in diameter, 10 patients (T3a) had multifocal tumors (<3 lesions), 22 patients were T3b of whom 13 patients had solitary, 5 had multifocal tumors (≤4 tumor lesions), and 4 had >4 tumor nodules). In 28/313 (8.9%) patients with CLIP4, 14 were solitary, 5 were multifocal tumors (≤4 tumor lesions), and 9 had >4 tumor nodules. In 12/313 (3.8%) patients with CLIP5, 9 were solitary, 1 was a multifocal tumor lesion (≤4 tumor lesions), and 2 had >4 tumor nodules. In 18/313 patients (5.8%) at stage T4 with a median tumor size of 6.64 cm (±3.846) in diameter, 14 were solitary and 4 were multifocal tumors (≤3 lesions).

RETRACTED

**Table 3:** The pathologic characteristics of HCC patients based on CLIP and TNM staging systems.

Variables	N (%)	Tumot Size (cm)		Portal vein or hepatic vein invasion	Lymph node invasion
		Mean	Std. Deviation		
T1	178(56.9)	4.16	2.329	0 (0.0)	0 (0.0)
T2	85(27.2)	3.11	1.442	0 (0.0)	0 (0.0)
T3 (3a+3b)	32(10.2)	7.58	3.234	22 (68.7)	0 (0.0)
T4	18(5.8)	6.64	3.846	6(33.3)	18(100.0)
CLIP criteria					
CLIP 0	54(17.3)	3.63	1.354	0 (0.0)	1(5.6)
CLIP 1	86(27.5)	3.57	1.637	0 (0.0)	4(22.2)
CLIP 2	82(26.2)	4.00	2.410	0 (0.0)	4(22.2)
CLIP 3	51(16.3)	4.74	3.052	8(15.7)	3(16.7)
CLIP 4	28(8.9)	7.12	3.710	10(35.7)	5(27.7)
CLIP 5	12(3.8)	7.90	4.025	10(83.3)	1 (5.6)

The majority of patients (89.1%) had moderately differentiated HCC (histologic grade II), while 13 (4.2%) had well-differentiated (histologic grade I), and 21 (6.7%) had poorly differentiated HCC (histologic grade III). Vascular invasion was present in 41 patients (13.1%). Among these patients, 28 had invasion of the main portal vein, portal vein branch or hepatic vein (22 patients with T3b and 6 patients with T4, of which 8 patients were CLIP3, 10 patients were CLIP4, and 10 patients were CLIP5 (Table 3). Thirteen patients had only microvascular invasions. These data, including a case of perihepatic lymph node invasion detected by a pathologist after LT, are shown in Table 3.

The overall and tumor recurrence-free survival rates of HCC patients based on the TNM classification (T1-4) and the CLIP tumor staging systems are shown in Table 4. The Kaplan-Meier curves showed clearly different survival rates for patients scored according to the CLIP 1–5, and T1–4 staging systems with high statistical significance (P<0.05) in all cases. Moreover, there were highly statistically differences in the overall survival or tumor recurrence-free survival between T2 and T3 patients (P<0.001 in both cases). The overall 1-, 3-, and 5-year survival rates for the patients with T2 were 96%, 90% and 81%, respectively, while patients with T3 were 51%, 34% and 26% for the 1-, 3-, and 5-year survival rates, respectively. For patients with CLIP 3, the 1-, 3-, and 5-year survival rates were 86%, 76%,and 71%, respectively.

RETRACTED

**Table 4:** Univariate analysis of patient overall survival and recurrence-free survival based on the TNM and CLIP staging systems.

Variables	Overall survival rate (%)			P-value	Tumor recurrence-free survival rate (%)			P-value
	1 year	3 years	5 years		1 year	3 years	5 years	
T1	95	92	90		93	91	91	
T2	96	90	81	0.023	83	79	79	0.018
T3 (3a+3b)	51	34	26	0.000	33	24	24	0.000
T4	72	50	44	0.000	48	35	35	0.000
CLIP criteria								
CLIP 0	98	92	90		92	92	90	
CLIP 1	100	98	94	0.304	96	96	96	0.350
CLIP 2	93	85	77	0.012	81	72	72	0.012
CLIP 3	84	76	71	0.000	76	70	70	0.008
CLIP 4	67	60	53	0.000	54	54	54	0.000
CLIP 5	40	20	20	0.000	22	22	22	0.000

### Patient survival and recurrence

During follow up, 86/313 patients (27.5%) died. Of the 86 patients, 70 (81.3%) died from tumor recurrence, and 16 (21.6%) died from other causes (1 case of sepsis, 3 of pulmonary infection, 2 of liver failure from rejection, 4 of liver failure from biliary passage complication, 1 of recurrent hepatitis, 1 of graft versus host disease [GVHD], 1 of acute myocardial infarction, 1 of cerebrovascular accident, 1 of hemorrhagic shock, and 1 case had a traffic accident). Recurrence of HCC was the most common cause of death after LT.

The median tumor recurrence-free survival time of the 313 patients was 59 months. Of the 313 patients, univariate analysis showed that the overall 1-, 3-, - and 5 -year survival rates were 90%, 84%, and 78.3%, respectively, and the 1-, 3-, and 5- -year tumor recurrence-free survival rates were 82%, 78% and 78%, respectively. Patients in the Milan group or the Milan-UCSF group had good survival after LT, with 3- and 5-year overall survival rates of 95% and, 91% or 91% and 79%, respectively.

There was HCC recurrence in 78/313 patients (24.9%) with a median time to recurrence of 11 months (range, 1–49). With regards to the sites of the first tumor recurrence, 28/78 cases (35.9%) were intrahepatic, 32/78 cases (41.0%) were in the lung, 5/78 (6.4%) cases were in the bone, 2/78 (2.6%) cases in the head, 3/78 (3.8%) were in the adrenal gland, 1/78 (1.3%) cases were in the peritoneum (0.1%), and 5/78 of the patients (6.4%) had both intrahepatic and extrahepatic recurrence, as well as 2 patients with new-onset malignant tumor in the stomach or esophagus over 3 years after LT.

RETRACTED

Postoperative HCC therapy was given to 54/313 patients (17.3%) who were diagnosed with tumor recurrence during LT follow-up. Therapy consisted of radiotherapy (18 cases, 33.3%), transarterial chemoembolization (3 cases, 5.5%), percutaneous ablations (4 cases, 7.4%), and reoperation (14 cases: 10 resection [18.5%] and 4 LT [7.4%]), as well as combinations of 2 or 3 HCC therapies (15 cases, 27.8%).

### Univariate analysis of prognostic factors for overall survival and tumor recurrence-free survival

Prognostic factors for overall survival identified through univariate analysis are reported in Table 5. Among the pre-LT factors, tumor size (>5 cm), tumor number (≥2), poor tumor differentiation, vascular invasion and lymph node invasion, high serum AFP level, and poor liver function (ALT and AST levels) were all significant risk factors affecting overall survival post-LT. Patients with serum AFP levels ≤1000 µg/L did better post-LT, with 1-, 3-, and 5-year overall survival rates of 94%, 80% and 80%, respectively (P = 0.011) compared to patients with serum AFP levels >1000. Patients with ALT levels (<1N) did better post-LT, with 1-, 3-, and 5- year overall survival rates of 97%, 91%,and 86%, respectively (P = 0.004) compared to patients with ALT levels (>1N). In contrast, patients with AST levels (≥3N) were associated with poor overall survival post-LT, with 1-, 3-, and 5-year overall survival rates of 71%, 62%, and 60% (P = 0.000), respectively. All patients received antivirus treatment, and the HBV reinfection rate (6.4%) had a significant association with overall survival post-LT (P = 0.049).

**Table 5:** Univariate analysis of patient characteristics and overall survival risk factors.

Variables	Overall survival rate (%)				P-value
	1 year	3 years	5years	7years	
Gender					
Male	90	83	78	72	
Female	92	88	88	88	0.288
Age (year)					
≤50	89	82	81	76	
>50	91	95	76	70	0.605
HBeAg					
Negative	90	82	78	75	
Positive	90	86	79	68	0.807
HBV-DNA(×10^3^ IU/ml)					
<1	92	87	81	75	
>1	90	83	78	74	0.885
Child-Pugh score					
A	92	84	77	75	
B	87	84	82	73	0.901
C	92	84	76	73	0,929
ALT(IU/L)					
1N,	97	91	86	82	
≥1N,<2N	86	78	71	65	0.004
≥2N, <3N	84	81	73	73	0.112
≥3N	89	76	76	68	0.053
AST(IU/L)					
1N,	97	93	84	84	
≥1N,<2N	89	82	79	69	0.065
≥2N, <3N	93	86	80	75	0.376
≥3N	71	62	60	60	0.000
ALP(IU/L)					
1N,	95	88	81	75	
≥1N, <2N	82	77	74	71	0.233
≥2N	73	67	67	67	0.064
Tumor size (cm)					
≤3	97	90	86	80	
>3, ≤5	98	93	86	78	0.959
>5, ≤7.5	83	72	66	66	0.006
>7.5	50	44	44	44	0.000
Number of tumor nodules					
Single	88	84	82	80	
2	96	82	64	47	0.010
3	100	100	100	100	0.096
4,	80	80	80	48	0.313
>4	91	77	71	71	0.390
Tumor differentiation					
I (well)	100	100	100	100	
II (moderate)	90	84	79	73	0.051
III (poor)	77	68	60,	60,	0.013
Serum AFP level (ng/ml)					
≤500	94	88	83	77	
500–1000	94	80	80	80	0.778
1000–2000	74	70	56	56	0.011
2000–5000	73	60	60	60	0.023
≥5000	58	50	50	25	0.000
Venous invasion					
Absent	95	89	84	78	
Present	48	39	33	33	0.000
Lymph node invasion					
Absent	91	86	81	76	
Present	72	50	44	33	0.000
Pre-LT antitumor therapy					
Absent	50	32	29	29	
Present	95	88	80	75	0.000
Post-LT HBsAg reinfection					
Negative	90	83	80	77	
Positive	95	90	56	42	0.049
Rejection					
Absent	90	83	78	72	
Present	93	89	85	85	0.232

The prognostic factors for the 1-, 3-, 5- and 7-year tumor recurrence-free survival rates identified through univariate analysis are reported in Table 6. Based on the Log Rank and Kaplan-Meier analyses, tumor size (>5 cm) (Fig. 1A), tumor number (≥2) (Fig. 1B), the presence of vascular invasion (Fig. 1C), poor tumor differentiation (Fig. 1D), lymph node invasion (Fig. 1E), pre-LT high serum AFP level (>1000 ng/ml) (Fig. 1F), ALT (≥3N) and AST level (≥3N) (Fig. 1G) were all significantly associated with poor recurrence-free survival after LT. In addition, we observed that the post-LT HBV re-infection rate (P = 0.027) was significantly associated with tumor recurrence.

RETRACTED

**Figure 1:** Univariate analysis of factors affecting of tumor recurrence-free survival rates of HCC patients in the study: (A) tumor size, (B) tumor number, (C) vascular invasion, (D) tumor differentiation, (E) lymph node invasion, (F) pre-LT serum AFP level, (G) pre-LT Serum ALT levels, and (H) pre-LT Serum AST levels.

**Table 6:** Univariate analysis of patient characteristics and tumor recurrence-free survival risk factors.

Variables	Tumor recurrence-free survival rate (%)				P-value
	1 year	3 years	5years	7years	
Gender					
Male	88	88	88,	88	
Female	81	78	77,	75	0.254
Age (year)					
≤50	82	80	80,	77	
>50	82	77	76,	75	0.663
HBeAg					
Negative	82	79	78	76	
Positive	82	78	78,	75	0.916
HBV-DNA(×10^3^ IU/ml)					
<1	84	79	79,	74	
>1	82	79	79,	77	0.939
Child-Pugh score					
A	81	79	78,	74	
B	83	79	79,	77	0.890
C	83	76	76	76	0.885
ALT(IU/L)					
1N,	87	86	86,	86	
≥1N, <2N	81	72	71,	63	0.002
≥2N, <3N	78	75	75,	75	0.091
≥3N	70	70	70,	70	0.017
AST(IU/L)					
1N,	90	89	88,	81	
≥1N, <2N	82	76	76,	74	0.034
≥2N, <3N	84	78	78,	78	0.207
≥3N	62	59	59,	59	0.000
ALP(IU/L)					
1N,	86	81	81,	77	
≥1N, <2N	75	74	72,	72	0.129
≥2N	69	69	69,	69	0.104
Tumor size (cm)					
≤3	86	86	86,	86	
>3, ≤5	91	85	85,	83	0.078
>5, ≤7.5	75	69	66,	57	0.006
>7.5	44	44	44,	44	0.000
Number of tumor nodules					
Single	84	82	82,	80	
2	71	63	63,	52	0.004
3	100	100	100,	100	0.088
4,	60	60	60,	60	0.268
>4	77	72	72,	72	0.357
Tumor differentiation					
I (well)	100	100	100,	100	
II (moderate)	82	79	78,	76	0.051
III (poor)	73	62	62	0	0.013
Serum AFP level (ng/ml)					
≤500	87	83	83,	80	
500–1000	88	80	80,	80	0.941
1000–2000	61	61	61,	61	0.005
2000–5000	56	56	56,	56	0.006
≥5000	42	42	42,	42	0.000
Venous invasion					
Absent	88	84	84,	81	
Present	36	32	32,	32	0.000
Lymph node invasion					
Absent	84	81	81,	78	
Present	48	35	35,	35	0.000
Pre-LT antitumor therapy					
Absent	33	27	27,	27	
Present	84	80	79,	79	0.000
Post-LT HBsAg reinfection					
Negative	82	80	80,	77	
Positive	80	53	53,	53	0.027
Rejection					
Absent	81	78	77,	75	
Present	89	86	86,	86	0.281

However, there was no significant difference in either the overall survival (P = 0.901, P = 0.929) or tumor recurrence-free survival (P = 0.890, P = 0.885) post-LT between Child-Pugh score A, B or C (Table 5 and 6). Remarkably, no significant difference in overall survival (P = 0.647) or tumor recurrence-free survival (P = 0.596) were shown between patients with >4 tumors and patients with ≤4 tumors.

RETRACTED

### Independent prognostic factors for overall survival and tumor recurrence-free survival

Independent prognostic factors for overall survival identified through multivariate analysis are reported in Table 7. Multivariate analysis showed that tumor size >7.5 cm (P = 0.001, hazard ratio [HR] = 3.528; 95% confidence interval [CI]: 1.717–7.246), tumor number >1 (P = 0.004, HR = 2.196; CI 1.285–3.752), the presence of vascular invasion (P = 0.002, HR = 2.740; CI 1.450–5.177), the pre-LT serum AFP level ≥1000 ng/ml (P = 0.010, HR = 2.083; CI: 1.192–3.641) and an AST level ≥120 IU/L (P = 0.044, HR = 2.061; CI:1.021–4.160) were all independent predictors of poor survival post-LT. However, the ALT level was not an independent predictor for overall survival post-LT by multivariate analysis.

**Table 7:** Multivariate analysis of patient characteristics and overall survival risk factors.

Variables	B	SE	Wald	Sig.	Exp(B)	95.0% CI for Exp(B)	
						Lower	Upper
Age(≤50 v>50 y)	0.178	0.248	0.517	0.472	1.195	0.735	1.943
Venous invasion	1.008	0.325	9.637	0.002	2.740	1.450	5.177
Lymph node invasion	0.623	0.391	2.536	0.111	1.864	0.866	4.010
Pre-LT tumor therapy	−0.643	0.293	4.831	0.028	0.526	0.296	0.933
Tumor size (≤7.5 v>7.5 cm)	1.261	0.367	11.783	0.001	3.528	1.717	7.246
Tumor number (1 v>1)	0.786	0.273	8.279	0.004	2.196	1.285	3.752
AFP(<1000 v ≥1000 ng/ml)	0.734	0.285	6.642	0.010	2.083	1.192	3.641
ALT (≤40 v>40 IU/L)	−0.055	0.410	0.018	0.893	0.946	0.424	2.114
AST (<120 v ≥120 IU/L)	0.723	0.358	4.071	0.044	2.061	1.021	4.160

Independent prognostic factors for recurrence-free survival identified through multivariate analysis are reported in Table 8. Multivariate analysis showed that independent predictors of poor recurrence-free survival were tumor size >7.5 cm (P = 0.001, HR = 3.309; CI 1.607–6.814), a tumor number >1 (P = 0.005, HR = 2.154; CI 1.260–3.682), the presence of vascular invasion (P = 0.001, HR = 2.788; CI 1.496–5.196), and a pre-LT serum AFP level ≥1000 ng/ml (P = 0.009, HR = 2.094; CI 1.200–3.653). The Cox proportional hazard model also showed that the higher the tumor size or the pre-LT serum AFP level, the higher the risk ratio, and there was no the relation with tumor number. Patients with pre-LT antitumor therapy had a significantly lower likelihood of recurrence-free survival (P = 0.011, HR = 0.484; CI 0.277–0.845).

RETRACTED

**Table 8:** Multivariate analysis of patient characteristics and tumor recurrence-free survival risk factors.

Variables	B	SE	Wald	Sig.	Exp(B)	95.0% CI for Exp(B)	
						Lower	Upper
Age (≤50 v>50 y)	0.230	0.252	0.834	0.361	1.258	0.769	2.060
Venous invasion	1.025	0.318	10.417	0.001	2.788	1.496	5.196
Lymph node invasion	0.605	0.388	2.431	0.119	1.831	0.856	3.918
Pre-LT tumor therapy	−0.611	0.293	4.360	0.037	0.543	0.306	0.963
Tumor size (≤7.5 v>7.5 cm)	1.197	0.369	10.537	0.001	3.309	1.607	6.814
Tumor number (1 v>1)	0.767	0.274	7.865	0.005	2.154	1.260	3.682
AFP(<1000 v ≥1000 ng/ml)	0.739	0.284	6.773	0.009	2.094	1.200	3.653
ALT (≤40 v>40 IU/L)	0.312	0.304	1.052	0.305	1.366	0.753	2.477
AST (<120 v ≥120 IU/L)	0.587	0.308	3.627	0.057	1.799	0.983	3.291

### Pre-LT antitumor therapy

Among 313 patients, univariate analysis showed that the overall survival (P = 0.000) and recurrence-free survival rates (P = 0.000) of patients with pre-LT antitumor therapy were better than those of patients with no pre-therapy for HCC (Tables 5 and 6; Fig. 1H). Multivariate analysis (Tables 7 and 8) showed that pre-LT antitumor therapy was an independent predictor of good survival (P = 0.028, HR = 0.526; CI: 0.296–0.933) and recurrence-free survival (P = 0.037, HR = 0.543; CI: 0.306–0.963),

Among those in the exceeding UCSF criteria group, statistical analysis showed that 38 patients with pre-LT antitumor therapy had a better overall survival (P = 0.000) and recurrence-free survival rates (P = 0.000, Fig. 2) than those of patients without pre-LT antitumor therapy for HCC. The 1-, 3-, and 5-year overall survival rates of patients who exceeded the UCSF criteria with pre-LT antitumor therapy were 92%, 87% and 83%, respectively, while patients without pre-LT antitumor therapy had rates of 56%, 38% and 35%,, respectively.

**Figure 2:** Kaplan-Meier analysis of the recurrence-free survival rates of patients with and without antitumor therapy pre-LT in the exceeding UCSF group.

RETRACTED

### Proposed Modified Tumor Staging Classification

Based on our observations, we defined an expanded set of criteria for HCC patients with HBV- cirrhosis that was associated with excellent survival after LT. These criteria included: solitary tumor <7.5 cm, ≤4 nodules with the largest lesion ≤6.5 cm or multiple nodules (>4) with the largest lesion ≤3 cm, and a pre-LT serum AFP level ≤1000 ng/ml and a AST level <120 IU/L (3N) without vascular invasion of the major portal vein branches or lymph node metastasis. Among 313 patients with HCC, statistical analysis showed that the 3- and 5-year overall survival rates of patients who fit the revised criteria were 95% and 90%, respectively, essentially identical to the survival rates in patients who fit the Milan or UCSF criteria in this study, with 5-year overall survival of 91% or 88%, respectively.

Among the exceeding UCSF criteria group, the Log Rank analysis showed that 19 patients fit our revised criteria, and all of them had a good overall survival (P = 0.002) and recurrence-free survival (P = 0.001), with 5-year overall survival and recurrence-free survival rates of 89% and 82%, respectively (Table 9). Patients who exceeded our revised criteria had 5-year overall survival and recurrence-free survival rates of 47%, and 45%, respectively (Fig. 3). Eight of the 19 patients had pre-LT antitumor therapy. There were no significant differences in overall survival post-LT between patients who fit our revised criteria and patients in the Milan group (P = 0.444) or the Milan-UCSF group (P = 0.866) (Table 9).

**Figure 3:** Kaplan-Meier analysis of the overall survival rates of patients who were fit and unfit for the revised criteria in the exceeding UCSF group.

**Table 9:** The overall survival and recurrence-free survival rates of patients who fit the Milan, Milan-UCSF, and revised criteria in the exceeding UCSF group.

Variables	Overall survival rate (%)			P-value	Tumor recurrence-free survival rate (%)			P-value
	1 year	3 years	5 years		1 year	3 years	5 years	
Fit revised criteria	100	89	89		94	82	82	
Fit Milan	98	95	91	0.444	93	90	89	0.484
unfit Milan, but fit UCSF	95	90	79	0.866	88	83	80	0.753

## Discussion

The prognostic assessment of HCC patients with HBV-cirrhosis is complicated by factors such as liver function, HBV infection, and tumor characteristics [5]. It is currently known that survival and recurrence post-LT are affected by tumor characteristics such as tumor size, tumor number, differentiation, vascular invasion, lymph node metastasis, and pre-LT serum AFP levels [14], [18], [19]. However, these risk factors have not been adequately assessed in studies with large enough sample sizes, and there is no universally accepted suitable selection policy for LT in HCC with HBV- cirrhosis. The present study addressed this deficiency by performing a stratified analysis of 313 HCC patients with HBV -cirrhosis who underwent LT with antiviral therapy.

RETRACTED

Univariate analysis and multivariate analysis in the current study showed that independent predictors of tumor recurrence and poor LT outcome for HCC patients with HBV-associated cirrhosis were tumor size >7.5 cm, tumor number >1, the presence of vascular and lymph node invasion, and pre-LT serum AFP levels ≥1000 ng/ml, and AST levels ≥120 IU/L. In addition, pre-LT antitumor therapy remained a significant independent factor for survival, with a 5-year survival of 80% with pre-LT therapy. This finding is consistent with previous reports [33], [34] and supported the use of downstaging therapy pre-LT for HCC patients with HBV-associated cirrhosis. We suggest that the important predictors in determining outcome post-LT for HCC patients with HBV-associated cirrhosis are not just the pathologic tumor factors, but also the AFP levels, liver function levels and pre-LT antitumor therapy. The prevailing criteria such as Milan and UCSF are limited for HCC patients when only the factors of tumor size and tumor number are included. Therefore, we recommend expanding the selection criteria for LT of HCC patients with HBV-associated cirrhosis to include pre-LT therapy for HCC.

In the current study, the overall survival rates for the 313 patients after LT were 90%, 84% and 78.3% at 1, 3, and 5 years, respectively. It is generally accepted that adjuvant antiviral treatment for LT patients with HBV-related HCC can prevent HBV reinfection [25], [35]–[37]. In the present study, comprehensive antiviral prophylaxis with hepatitis B immune globulins (HBIg) and lamivudine, adefovir or entecavir were given to all the patients, of whom only 6.40% had HBV reinfection after LT. This result is similar to other reports [22], [38]–[39], and indicates that antiviral prophylaxis can prevent HBV reinfection and that antiviral therapy is effective in improving survival of LT patients with HCC.

It was reported that the outcome for patients with advanced HCC is related not only to tumor stage, but also to the extent of liver dysfunction [20]–[23]. Fidel-David et al [23] showed that the TNM (sixth edition) classification system alone was not useful for predicting overall survival, but CLIP staging systems were good informative staging systems in predicting survival in patients with advanced HCC. Five prognostic strata were defined according to a score derived from the analysis of variables related to cirrhosis (Child-Pugh score), tumor morphology, AFP level, and portal vein thrombosis. In this study, the 5-year survival rates of patients in the current study with CLIP 0–2 or stage T1–2 were similar to the survival rates of Milan criteria reported by Mazzaferro et al. [8] (83% at 4 years) for similar tumor stages. However, for patients who exceeded the Milan or UCSF criteria, there were 25% patients with CLIP 1–2, and 32.6% patients with CLIP 3, while there were 54.3% patients with stage T1–2. The overall survival rates of 1-, 3- and 5-years for the patients with CLIP3 were 86%, 76% and 71%, respectively, while for the patients with stage T3, the overall survival rates were 51%, 34% and 26%, respectively. The result showed that HCC patients with CLIP >2 may still have a favorable outcome after LT.

RETRACTED

Remarkably, our results also showed that there were no significant differences in the overall survival or recurrence between patients with >4 tumors lesions and patients with ≤4 tumors lesions. Furthermore, our results showed that HCC patients with stage T2 had a good overall survival, with 81% 5-year overall survival rates versus 26% in patients with stage T3a. According to the TNM staging systems (UICC/AJCC, 2010), patients who had multiple tumors, any of which were ≤5 cm in diameter, were considered to be at stageT2, while patients with multiple tumors, any of which are >5 cm, were considered to be at stage T3a. Therefore, we recommend expanding the selection criteria for LT of HCC patients with HBV-associated cirrhosis to include multifocal tumors (>3) with a limit in tumor size based on T2.

Our study also suggests that excellent survival can be achieved in HCC patients with CLIP3 and T2 who meet our proposed criteria: solitary tumor ≤7.5 cm, ≤4 multifocal nodules with the largest lesion ≤5 cm and a total tumor diameter ≤10 cm or multiple nodules with the largest lesion ≤3 cm, and a pre-LT serum AFP level <1000 ng/ml and a AST level <120 IU/L without vascular invasion of the major portal vein branches or lymph node metastasis. In the study, HCC patients who fit our revised criteria, but exceeding UCSF criteria, had survival rates of 89% at 5 years, and did better than those patients who exceeded our revised criteria, with survival rates of 47% at 5-years Moreover, the overall survival rates in patients who fit our revised criteria were similar to that in patients who fit the Milan or UCSF criteria (91% or 79%).

There have been several previous studies that have provided some evidence for predicting survival outcomes after LT [18]–[20], [33], [34], [40], [41]. Except for several reports on small HCC with good survival using criteria such as Milan [8] or UCSF [14], et al. Marsh et al [42] reported that a subgroup of PT4 patients with 4 or more nodules, none greater than 3 cm, had a 5-year tumor-free survival rate of 80%. However, Tan et al. [43] reported that patients with HCC less than 8 cm (multifocal in 10 patients) who underwent LT had disease-free survival rates of 80% and 63% at 1 and 3 years, respectively. McPeake et al. [44] showed less favorable results for patients with larger or multifocal tumors. The limitation of their results might be due to a lack of detailed information on the size and number of lesions in the multifocal HCC, as well as on the pre-LT AFP levels, liver function levels and antitumor therapy pre-LT.

RETRACTED

ALT and AST levels in patients with chronic liver disease are considered markers of inflammation that reflect the etiopathogenetic mechanism of hepatocyte necrosis [45], while the Child-Pugh score is considered an index of liver cirrhosis that reflects the severity of the clinical condition [46], [47]. When liver cells are damaged or dying, ALT and AST leak into the bloodstream. The resulting presence of these enzymes in serum is a clinical expression of a biologic activity of multicentric carcinogenesis [48]. Some reports have shown that high AST is an accurate predictor of tumor recurrence or poor outcome [45], [49]. High AST levels are predictors of recurrence because inflammation in the liver can stimulate production of some adhesion molecules on cancer cells in the remnant liver, and cause postoperative recurrence [49]. The current study demonstrated that pre-LT AST ≥3N levels were independent predictors of poor outcome in univariate analyses and were shown to be sensitive predictors of prognosis for LT in HCC patients with HBV-associated cirrhosis. However, Child-Pugh scores were not shown to be significant predictors of survival by univariate and multivariate analyses. The findings can be explained by the fact that repeated and severe inflammation and cellular necrosis enhance proliferation of HBV, as well as accelerate the development of HCC and the formation of micro-metastases by increasing the rate of random mutations. In addition, changes of enzymes and proteins in biochemical reactions of tumor cells often predict tumor development and progression [50]. Thus, based on the univariate and multivariate analyses, AST (<3N) as a significant predictor with an 80% 5-year overall survival rate was included in the expanded criteria in this study. Fidel-David et al [23], reported that AST is an independent prognostic factors for the overall survival of advanced HCC. We believe that the administration of adjuvant anti-inflammatory therapy with the appropriate anti-HBV treatment may improve AST levels.

RETRACTED

In addition, among those patients who exceeded UCSF criteria in this study, the majority of HCC patients received chemoembolization or combined with percutaneous ablations therapy for downstaging of tumors before LT. Those patients with pre-LT antitumor therapy had a better overall survival rate at 5-year (83%) than that of patients without pre-LT antitumor therapy (35%). This finding suggest that it is necessary to widely use antitumor therapy pre-LT for downstaging of tumors and to decrease the risk of tumor dissemination in HCC patients who exceed UCSF criteria during the increased waiting time for LT. From the results of the current study, this procedure did not influence the effect of operation in HCC patients with cirrhosis pre-LT whose hepatic function might have been damaged by chemoembolization or combined with percutaneous ablations therapy. Thus, our results support the use of pre-LT antitumor therapy in expanding the selection criteria to offer the potential benefit of LT to some advanced HCC patients with HBV-associated cirrhosis who would otherwise be excluded from LT.

Our results appear to differ from several previous studies reporting worse survival after LT for patients with solitary tumors over 6.5 cm or patients with 3 multifocal tumors of sizes >4.5 cm. Furthermore, the TNM stage needs to be precisely evaluated by pathologists. However, it is sometimes impossible to obtain clear-cut tumor characteristics preoperatively without a biopsy of the lesion which can introduce risk of tumor seeding along the biopsy tract by liver biopsy. The prevailing criteria such as Milan and UCSF are limited for predicting post-LT overcomes because they only include factors such as tumor size and tumor number.

In conclusion, we focused on cut-offs for tumor burden and re-calculated the statistics based on the results of using expanded criteria according to CLIP and TNM. We propose the adaption of expanded selection criteria for HCC patients with HBV-associated cirrhosis pre-LT: solitary tumor ≤7.5 cm, ≤4 multifocal nodules with the largest lesion ≤5 cm and a total tumor diameter ≤10 cm or more nodules with the largest lesion ≤3 cm, and a pre-LT serum AFP level ≤1000 ng/ml and a AST level <120 IU/L without vascular invasion of the major portal vein branches or lymph node metastasis. Such expanded selection criteria combined with antiviral prophylaxis and pre-LT therapy for HCC and inflammation may be a rational strategy to prolong survival after LT for HCC patients with HBV-associated cirrhosis. Randomized studies with larger sample sizes are needed to further evaluate the effect of these expanded selection criteria.
